# Research on the Protection of Extensor and Flexor Muscles in the Waist and Back of Competitive Athletes

**DOI:** 10.1155/2022/7378953

**Published:** 2022-07-04

**Authors:** Xuedou Yu, Ligang Ma, Ruihua He, Jian Zhao, Shanshan Wang

**Affiliations:** ^1^Hebei University of Engineering, Handan, 056038 Heibei, China; ^2^Capital University of Physical Education and Sports, Beijing 100191, China

## Abstract

In the past, in the study of special sports quality of heavy antagonistic sports events, the study of strength quality training was emphasized. The transformation of athletes' strength quality to special strength was highlighted, and the special exercises which tended to be consistent with the characteristics of wrestling events were added. However, in competition and training, athletes' spine bears a heavy load. Long-term static contraction of lumbar muscles can lead to excessive local load and injury of lumbar muscles. In this paper, the test results of athletes' joints are analyzed, and the waist protection scheme for athletes' strength training is obtained. First of all, solve the problem of athletes' action mode and improve athletes' muscle endurance. All special sports quality evaluation can reach a good level. Then, enhance athletes' explosive power. Thus, all special sports quality evaluations can reach an excellent level. It is concluded that the waist and back are the key parts to support their participation in various sports, maintain body balance, and realize power transmission. Through the study, it is found that there are significant differences in the muscle strength indexes of the maximum strength of the waist and back of athletes of different levels, which fully proves the characteristics of the maximum strength of the waist and back. Through the test, we can understand the flexion and extension strength, range, speed, force, and flexion and extension ratio of athletes' joints and take timely optimization measures according to the test results to avoid sports injuries in training. It has a key guiding significance for the measurement, analysis, and evaluation of athletes' joint muscle strength, as well as rehabilitation training after injury and prevention of reinjury.

## 1. Introduction

Sports quality covers athletes' general sports quality and special sports quality. General sports quality can make athletes' basic abilities develop in a balanced way. Special sports quality emphasizes the development of special sports ability which tends to be consistent with special sports ability. Special sports quality and general sports quality complement each other [1]. The characteristics of heavy anticompetitive sports are to achieve the maximum explosive force in a state of high-intensity confrontation. Special strength is very important in the project. Different special strength exercises should be carried out in the training according to the reasonable matching of training measurement and intensity in the growth stage of athletes [2]. Athletes' strength training, based on the theory of the special strength model, combines with practice, clarifies the training load, and strictly requires the range, angle, and speed of training. The strength training action of heavy anticompetitive sports should be combined with the technical characteristics of the project so that the muscle contraction mode is consistent with the special force characteristics to achieve a better transformation effect [3].

Through the analysis of athletes' muscle strength, experts conclude that the phenomenon of “immobility” often occurs in competitions caused by the weakness of athletes' spinal extension strength [4]. The strength imbalance of flexors and extensors in the trunk and neck will directly affect the performance of athletes in the competition. The lumbar and back tissues of the human body are shown in Figure 1.

By studying the differences between the flexors and extensors, internal and external rotators, and left and right muscles of the trunk, knee, elbow, and shoulder of wrestlers, it is concluded that the flexors and extensors of wrestlers cannot develop in a balanced way [5]. Some experts used advanced instruments to test athletes' special technical power stage, main joint strength, and muscle dynamic function and concluded that athletes should improve their latissimus dorsi and erector spinae strength exercises to increase the central nervous system's intensive stimulation of antagonistic muscle. The peak torque of athletes' lumbar back muscle is larger than that of the knee joint, and the extensor is larger than the flexor. The difference between the extensor and flexor easily leads to insufficient strength for athletes and the failure to complete the action. With the increase in speed, the strength of athletes' lumbar back extensor muscle group decreases. Attention should be paid to the coordinated development of athletes' lumbar back flexion and extensor muscle group [6].

Athletes need to have the maximum strength, explosive strength, and static strength of the whole body. Martin (2019) pointed out in his research that in addition to the above three kinds of strength, athletes should also have sufficient training experience and flexibility. From this point of view, athletes with high single quality and ability cannot be very sure to win the competition, but excellent athletes must have many excellent qualities and abilities [7]. Owen et al. (2019) once found in the training monitoring of elite wrestlers that after four times a week of strength training for large muscle groups, the athletes all suffered from muscle injuries. After four times a week of training for small muscle groups, the athletes' muscle injuries were restored, so the alternation of the two training methods was put forward. At the same time, it is suggested to analyze the training methods of athletes in combination with the training monitoring video of athletes to evaluate the training results of athletes more objectively [8]. Mathew et al. have conducted relevant research on strength training, pointing out that barbell bench press, bench pull, and squat can effectively improve the maximum strength of athletes. The improvement of fast strength requires the combination of maximum strength training and muscle contraction speed training [9]. Goris et al. have studied the characteristics of upper limb joint muscle strength of wrestlers. Combining with the characteristics of wrestling, they found that many scoring movements in heavy antagonistic sports are completed by upper limb strength [10]. In the current research results, they are all single-joint studies on heavy antagonistic sports, lacking systematic studies on multijoint. Therefore, the test and analysis of multijoint muscle strength in heavy antagonism and the study of the relationship between joint strength have become the key development direction of sports discipline in the future.

This paper analyzes the test results of athletes' waist physical fitness index, obtains the waist protection scheme for athletes' strength training, and summarizes that the waist and back are the key parts to support them to participate in various sports, maintain body balance, and realize power transmission. Through the study, it is found that there are significant differences in the maximum strength of the waist and back of athletes at different levels, which fully proves the characteristics of the maximum strength of the waist and back.

The main innovations of this study are as follows:

1. Based on the theoretical level of systematic research, the ISOMED2000 muscle strength testing system was used to test the flexion and extension muscle strength of elite male athletes in active service at three speeds of 60°/s, 180°/s, and 300°/s. Under this background, the differences in joint strength among different levels of athletes were analyzed
2. The characteristics of muscle strength and the relationship between joints and muscles in this paper can straighten out the development of joints and muscle strength in heavy antagonistic sports and also provide some countermeasures and suggestions for athletes' targeted training
3. In view of the deficiency of the current research on a single joint, this paper combines the muscle strength characteristics of each joint to carry out in-depth research on multisite comprehensive force, starting from the shoulder joint, knee joint, elbow joint, and waist and back

## 2. Research Object and Method

### 2.1. The Research Object

In this paper, the characteristics of muscle strength of wrestlers in heavy antagonistic sports are taken as the research object, and the wrestlers in active service are taken as the test object. According to their personal best sports results, they are divided into national masters and first-class athletes. The level is 60-130 kg, and there are no acute injuries in the first three weeks of the test [11]. The indicators selected in this study are relative indicators, excluding the influence of athletes' weight, which is shown in Table 1.

### 2.2. Research Methods

1. Method of measurement

The ISOMed2000 multijoint isokinetic testing system equipment produced in Germany was used for testing [12].

Test joints include the shoulder, elbow, wrist, lumbodorsal muscles, hip, knee, and ankle. Test indicators refer to relative peak torque, relative average peak torque, relative average power, work fatigue index, flexion and extension torque ratio, height, weight, etc. [13].

Relative peak torque (PT) refers to the maximum torque output generated by contraction of muscles or muscle groups during exercise, representing the maximum muscle strength of muscles or muscle groups. It is an important index of the isokinetic test [14].

Relative average peak torque (AT) refers to the average torque output generated by the contraction of muscles or muscle groups during exercise, representing the average muscle strength of muscles or muscle groups [15].

The work fatigue index reflects the endurance level of joint muscles [16].

The flexion and extension moment ratio is the ratio of flexor and extensor moment of joint muscles, reflecting the coordination ability of muscles [17].

Test speed: test the relative peak torque, relative average peak torque, relative average power, work fatigue index, and flexion and extension torque ratio at three speeds of 60°/s, 180°/s, and 300°/s to reflect the muscle strength characteristics of the joint at different speeds [18].

Test process: before the formal warm-up, let the athletes carry out joint activities to make the body reach a good state to meet the test, and then, start the test machine to start the test. At the same time, it is necessary to measure the height, weight, and dimensional indicators of the upper and lower limbs of the athletes, record the basic information of the athletes, and input it into the test instrument [19].

(3) Mathematical statistics

The Excel software was used to count all the test results as a whole, and the SPSS 22.0 computer analysis software was adopted to process the test data. All the data were expressed by average + standard deviation. Athletes' related test data were compared by the independent *t*-test. The significant difference was *P* < 0.05, and the very significant difference was *P* < 0.01. To reduce the analysis error, the data is analyzed by relative value [20].

### 2.3. Technical Route

The technical research route of this paper is shown in Figure 2.

## 3. Evaluation of Waist Protection in Heavy Antagonism Events

### 3.1. Evaluation Results of Maximal Isometric Muscle Strength of the Lumbar Spine in All Directions

The evaluation results of lumbar muscle strength in all directions of subjects in the control group and experimental group before and after 5 weeks of intervention are shown in Table 2.

Before the intervention, there was no significant difference between the experimental group and the control group in the muscle strength of the lumbar spine in all directions (*P* > 0.05).

Lumbar flexion muscle strength within the group: compared with before intervention, after 5 weeks of intervention, there was no significant difference between the two groups (*P* > 0.05).

Lumbar anteflexion muscle strength between groups: before the intervention and 5 weeks after the intervention, there was no obvious difference in lumbar anteflexion muscle strength between the control group and the experimental group (*P* > 0.05).

Lumbar extensor muscle strength within the group: compared with before intervention, the lumbar extensor muscle strength of the subjects in the experimental group and the control group increased significantly after 5 weeks of intervention (*P* < 0.05).

Lumbar left flexor muscle strength within the group: compared with before intervention, the lumbar left flexor muscle strength of the subjects in the experimental group and the control group increased significantly after 5 weeks of intervention (*P* < 0.05).

### 3.2. Test Results of the TMG Muscle Function Status Analyzer

The evaluation results of left TMG indexes of subjects in the experimental group and control group before and after 5 weeks of intervention are shown in Table 3.

Before the intervention, there was no significant difference in left TMG indexes between the experimental group and the control group (*P* > 0.05).

Left Dm value within the group: after 5 weeks of intervention, the left Dm value of the experimental group decreased, but there was no significant difference (*P* > 0.05), while the left Dm value of the control group increased, but there was no significant difference (*P* > 0.05). There was no significant difference in the left Dm value between the experimental group and the control group before and after the intervention for 5 weeks (*P* > 0.05). The evaluation results of TMG indicators on the right side of the subjects in the experimental group and the control group before and after 5 weeks of intervention are shown in Table 4.

### 3.3. Results of the Evaluation of Waist and Back Muscle Endurance Plank Support Time

Before the intervention and after 5 weeks of intervention, the results of back muscle endurance plank support time of the subjects in the experimental group and the control group are shown in Table 5.

## 4. Analysis of the Waist Protection Scheme in Heavy Antagonism Sports Event

### 4.1. Evaluation and Analysis of Maximal Isometric Muscle Strength of the Lumbar Spine in All Directions

The results of this study are shown in Table 2 and Figure 3. Physical therapy can significantly improve the muscle strength of the waist and back with lumbar muscle strain.

After 5 weeks, the maximum isometric muscle strength of the experimental group increased by 52.42% in the extension direction, 41.40% in the left flexion direction, 40.37% in the right flexion direction, and 41.67% in left rotation direction. The maximum isometric muscle strength in the right rotation direction increased by 28.85%.

In the control group, the maximum isometric muscle strength increased by 25.60% in the extension direction, 27.87% in the left flexion direction, 36.70% in the left rotation direction, and 12.94% in right rotation direction.

Through the analysis of the factors affecting the maximum isometric muscle strength, after 5 weeks of intervention, the increase in the maximum isometric muscle strength of the two groups of subjects may be due to the treatment of fascia knife combined with infrared physiotherapy, which effectively alleviated the symptoms and dysfunction of low back pain and also eliminated the fear of pain and fear of exerting force, that is, on the basis of improving the symptoms of lumbar muscle strain. The subject's muscle function and performance improved. Five weeks later, compared with other groups, the mean value of maximum isometric muscle strength in all directions was significantly higher than that in the other two groups. The possible reason was that the treatment combined with infrared physiotherapy not only greatly alleviated the symptoms of low back pain and eliminated the fear of pain but also activated the deep muscles of the back, strengthened the core muscles of the back, and enhanced the spine. It can also significantly enhance the stability of the waist [21].

### 4.2. Test and Analysis of the TMG Muscle Function Status Analyzer

The results of this study are shown in Figure 4. Fascia knife combined with infrared physiotherapy can improve the functional status of muscles.

After 5 weeks of intervention, the mean Tc value of the right side decreased significantly (*P* < 0.05), and the relatively low Tc value indicated that the muscle contraction speed was faster and the contraction ability was stronger. To sum up, the infrared physiotherapy treatment can significantly reduce the Tc value of the right-back muscle, improve the contraction speed and contraction ability of the right-back muscle, and improve the functional status of the left-back muscle [22].

### 4.3. Evaluation and Analysis of Waist and Back Muscle Endurance Plank Support Time

In this experiment, the duration of maintaining standard plank support was used to measure the muscle endurance of the subjects' waist and back.

The results of this study are shown in Figure 5. The treatment with fascia knife combined with infrared physiotherapy and infrared physiotherapy can significantly improve the muscle endurance of lumbar and back muscles and the time endurance of plank support in patients with a lumbar muscle strain.

Compared with before intervention, after 5 weeks of intervention, the evaluation results of the plank support time of the back muscle endurance of the experimental group and the control group were significantly increased (*P* < 0.05). The average evaluation results of the plank support time of the back muscle endurance of the experimental group after 5 weeks increased by 56.66%. After 5 weeks, the mean value of muscle endurance flat support time increased by 90.55%, and the mean value of muscle endurance flat support time increased by 42.22% in the control group.

The results showed that after 5 weeks of intervention, there was a significant difference in the time of flat support between the two groups (*P* < 0.05), which showed that the treatment of infrared physiotherapy was higher than that of fascia knife combined with infrared physiotherapy. The time of flat support was higher than that of infrared physiotherapy. The reason for the increase in the duration of the plank in the experimental and control groups may be that the pain was relieved to a certain extent and the plank level was partially restored (not fully restored to the previous level), rather than that the subjects actually improved the time of the plank [23]. After 5 weeks, the time of back muscle endurance plank support was significantly longer than that of the experimental group (*P* < 0.05), which could activate the deep muscles of the back, enhance the strength of the core muscles of the back, enhance the endurance of the back muscles, and also significantly enhance the stability of the waist.

## 5. Conclusion

Through the study of heavy antagonism sports events, this paper analyzes the characteristics of lumbar muscle indexes of different athletes in the process of competition and training. The experimental comparative analysis was carried out on the recovery of waist and back under different interventions. The results showed that different schemes of treatment plus physiotherapy had good therapeutic effects on lumbar muscle strain. The main research contents were as follows:

1. There are significant differences in the maximum strength of elbow extensor muscle among different levels of athletes, which shows that the maximum strength plays an important role in the elbow joint. At the same time, there are obvious differences in the strength endurance of the elbow joint among different levels of athletes. Both strength endurance and maximum strength are of great significance to the elbow joint
2. The differences of shoulder muscle strength of male wrestlers in different levels of heavy antagonistic sports events mainly focus on the muscle strength indicators of fast strength and strength endurance
3. In different levels of athletes, the differences of knee muscle groups are mainly manifested in maximum strength, fast strength, and strength endurance, and the indexes of each muscle group will increase with the improvement of athletes' level

Through this experiment, it is proven that adding functional physical training on the basis of conventional training will promote the functional improvement of athletes' waist and back muscles and prevent the positive role of sports injury to achieve the purpose of improving the training effect.

There are also some shortcomings in this study. The number of subjects in this study is limited, which may have a slight impact on the accuracy of the experimental results. In future studies, the sample size should be increased to improve the accuracy of the experimental results.

## Figures and Tables

**Figure 1:** Musculature of the back.

**Figure 2:** Technical route.

**Figure 3:** Changes of muscle strength of lumbar vertebrae in different motion directions after intervention.

**Figure 4:** Changes in right TMG test data after intervention.

**Figure 5:** Changes of waist and back muscle endurance and plank support time after intervention.

**Table 1:** Basic information about test objects.

	Athlete	First-class athlete
Number of people *n*	7	15
Age	24.71 ± 5.29	19.8 ± 2.08
Training years (years)	13.05 ± 3.01	7.90 ± 2.83
Height (cm)	181.71 ± 8.56	182.35 ± 5.36

**Table 2:** Evaluation results of maximum isometric muscle strength of subjects in each movement direction of lumbodorsal muscles.

Groups	Comparison period	Forward bends (nm)	Stretch back (nm)	Left lateral flexion (nm)	Right lateral flexion (nm)	Left-handed (nm)	Right-handed (nm)
Control group	Before the intervention	115.4 ± 32.6	172.2 ± 76.3	103.2 ± 70.3	100.6 ± 50.3	62.3 ± 42.1	63.1 ± 42.5
	Intervention for 5 weeks	133.4 ± 28.2	198.6 ± 40.1	121.8 ± 43.8	115.7 ± 21.9	76.3 ± 24.6	76.9 ± 21.5
Experimental group	Before the intervention	118.6 ± 35.7	169.7 ± 63.8	112.8 ± 67.3	109.7 ± 63.7	60.8 ± 41.9	61.1 ± 39.7
	Intervention for 5 weeks	164.8 ± 20.7	213.8 ± 27.9	134.7 ± 26.8	131.7 ± 19.8	83.6 ± 19.7	85.9 ± 18.7

**Table 3:** Left TMG test results of subjects.

Groups		Tc (ms)	Tr (ms)	Dm (mm)
Control group	Before the intervention	20.5 ± 6.5	89.5 ± 70.6	3.1 ± 1.8
	Intervention after 5 weeks	23.7 ± 4.8	113.8 ± 43.5	3.4 ± 1.5
Experimental group	Before the intervention	20.6 ± 7.1	90.6 ± 72.4	3.0 ± 1.9
	Intervention after 5 weeks	25.6 ± 7.5	121.6 ± 56.7	3.6 ± 1.7

**Table 4:** TMG test results on the right side of subjects.

Groups		Tc (ms)	Tr (ms)	Dm (mm)
Control group	Before the intervention	18.6 ± 6.7	106.7 ± 45.6	2.1 ± 1.3
	Intervention for 5 weeks	20.6 ± 5.4	112.3 ± 42.9	2.3 ± 1.1
Experimental group	Before the intervention	19.5 ± 5.7	109.7 ± 50.7	2.2 ± 1.7
	Intervention for 5 weeks	23.7 ± 4.8	124.9 ± 43.8	2.5 ± 1.5

**Table 5:** Evaluation results of plank support time of subjects' waist and back muscle endurance.

Experimental stage	Control group (s)	Experimental group (s)
Before the intervention	60.7 ± 23.5	62.7 ± 30.4
Intervention after 5 weeks	78.6 ± 20.6	89.3 ± 28.1

## Data Availability

The data used to support the findings of this study are available from the corresponding author upon request.
